# Detecting COVID-19 Pneumonia over Fuzzy Image Enhancement on Computed Tomography Images

**DOI:** 10.1155/2022/1043299

**Published:** 2022-01-18

**Authors:** Ali Alzahrani, Md. Al-Amin Bhuiyan, Fahima Akhter

**Affiliations:** ^1^Department of Computer Engineering, King Faisal University, Hofuf 31982, Saudi Arabia; ^2^College of Applied Medical Sciences, King Faisal University, Hofuf 31982, Saudi Arabia

## Abstract

COVID-19 is the worst pandemic that has hit the globe in recent history, causing an increase in deaths. As a result of this pandemic, a number of research interests emerged in several fields such as medicine, health informatics, medical imaging, artificial intelligence and social sciences. Lung infection or pneumonia is the regular complication of COVID-19, and Reverse Transcription Polymerase Chain Reaction (RT-PCR) and computed tomography (CT) have played important roles to diagnose the disease. This research proposes an image enhancement method employing fuzzy expected value to improve the quality of the image for the detection of COVID-19 pneumonia. The principal objective of this research is to detect COVID-19 in patients using CT scan images collected from different sources, which include patients suffering from pneumonia and healthy people. The method is based on fuzzy histogram equalization and is organized with the improvement of the image contrast using fuzzy normalized histogram of the image. The effectiveness of the algorithm has been justified over several experiments on different features of CT images of lung for COVID-19 patients, like Ground-Glass Opacity (GGO), crazy paving, and consolidation. Experimental investigations indicate that among the 254 patients, 81.89% had features on both lungs; 9.5% on the left lung; and 10.24% on the right lung. The predominantly affected lobe was the right lower lobe (79.53%).

## 1. Introduction

On December 31, 2019, the World Health Organization (WHO) released a statement that numerous cases of viral pneumonia with an unidentified cause had emerged in Wuhan, Hubei Province, China. On January 7, 2020, scientific research institutions in China confirmed that the viral pneumonia was caused by a novel coronavirus [1]. On February 11, 2020, the novel coronavirus was designated as severe acute respiratory syndrome coronavirus 2 (SARS-CoV-2) by the International Committee on Taxonomy of Viruses [2], and the disease caused by SARS-CoV-2 was termed “coronavirus disease 2019 (COVID-19)” by the WHO [3, 4]. The disease rapidly spread globally and became a pandemic. The scope of this ongoing pandemic was increasing exponentially while the world was struggling with a third wave of transmissions and many countries were trying to control the situation by intermittent lockdowns. Since then, the pandemic has had devastating effects on daily lives, public health, education, and economies. As of May 27, 2021, the number of confirmed cases was 167,492,769, including 3,482,907 deaths, with a mortality rate as mentioned on the WHO website [5]. The rapid spread of the disease has strained health-care systems worldwide because of shortages of essential protective equipment and health-care professionals along with unavailability of diagnostic kits and facilities. Therefore, quick identification of patients with COVID-19 is important for immediate management of patients and rapid isolation of patients to standstill the consequence of contamination [6].

Since COVID-19 is a highly communicable disease that causes inflammation in the respiratory system, the only effective way to control this spreading of infection is by rapid investigation of the population and isolation of the infected individuals. At present, the standard method for diagnosing COVID-19 is a positive outcome in nucleic acid testing (NAT) using reverse- transcription polymerase-chain-reaction (RT-PCR). This investigation provides high specificity, but low sensitivity [7]. Therefore, chest CT has turned into a precarious diagnostic procedure for COVID-19 manifestations since the affected lungs features can be detected by investigating radiological images of patients, even though negative results are obtained in RT-PCR test. Chest CT scans enable radiologists to understand the disease by providing a visual indicator of coronavirus infection and to determine the extent of the lesions, which supports accurate observations of changes. This motivated to the enhancement of CT imaging; and the investigation results have demonstrated that COVID-19 infected patients are detected more precisely using chest radiography images than other diagnostic techniques. The accurate and quick detection of COVID-19 assumed cases play a vital role in well-timed quarantine and remedial action.

A fair amount of research work has already been published in the literature on clinical manifestations and epidemiological evidences for COVID-19. Fang et al. [8] found that the sensitivity of CT (98%) was significantly higher than that of RT-PCR (71%) in diagnosing COVID-19 infected patients. Hani et al. [9] deliberated the clinical characteristic features of lung CT images for COVID-19 pneumonia and highlighted the chief diagnosis. They analysed the chronological CT images for their alterations during follow-up and tried to determine the clues for their detection. Bernheim et al. [10] presented a surveying study on chest CT images from indicative patients infected by coronavirus disease COVID-19 from different hospitals of China during January and February 2020. They studied for typical CT outcomes in association with the time between symptom inception and the first CT scan. The trademarks of COVID-19 contamination on images were bilateral and peripheral GGO and consolidative pulmonary opacities. At a longer interval from the commencement of COVID-19 indications, CT symptoms had been more persistent, besides consolidation, crazy paving, air bronchogram, pleural effusion, lung immersion, mediastinal lymphadenopathy, and reverse halo sign. Li et al. [11] made a surveying study with patients infected by coronavirus COVID-19 from different regions of Wuhan, China. They investigated the patients' usual clinical manifestations, disease symptoms, and evolvement features of chest CT images. They identified lesions in the peripheral lung, patchy GGOs, and consolidation. Wang et al. [12] presented a retrospective study on patients' epidemiological and radiological behaviour of COVID-19 in Hubei Province in China. They identified lung CT abnormalities and analysed the clinical and radiological features of the patients.

Numerous AI applications such as machine learning, pattern recognition, and image processing tools are efficiently employed to identify and predict COVID-19 infections and recommend a suitable response to shrink the spread and impact of the virus [13–16]. Wang et al. [17] proposed a supervised deep learning method employing 3D CT for COVID-19 detection and lesion segmentation. They localized the lung area employing a pre-trained deep neural network for the prediction of the probability of COVID-19 contamination. Kang et al. [18] presented a computer aided identification for COVID-19 through multi-view representation machine learning algorithm. They made multi-feature extraction from multiple views of CT images and trained a unified latent illustration for diagnosis. With the aim of representing the multi-features of lung CT images at different viewing conditions, they expressed the latent representations for training multiple aspects of COVID-19 lung CT image features. Waheed et al. [19] proposed a method to develop synthetic chest X-ray images by designing an Auxilary Classifier Generative Adversarial network (AGGAN) based model named CovidGAN. They enhanced the convolutional network model and arranged a deep learning strategy on the chest X-ray images for corona virus detection. They improved the performance of traditional convolutional neural network by employing synthetic images generated from CovidGAN.

Shorfuzzaman and Hossain [20] have developed a deep meta-learning based AI algorithm to augment the recognition of COVID-19 over chest X-ray (CXR) imaging. They addressed a synergistic method to incorporate a contrastive learning strategy with an adjusted trained ConvNet coder. To influence the unbiased feature representations and control a Siamese network for the final classification of COVID-19 features, they employed the Convnet architecture. The effectiveness of their approach has been endorsed employing two widely available datasets containing images from ordinary COVID-19 and those with COVID-19 complicated by pneumonia. Zhou et al. [21] proposed a UNet model for detecting coronavirus employing chest CT scan imaging. They investigated lung images over 106 patients as model training and evaluated their classification model. They claimed that the performance of their experiments was quite reasonable considering the time constraint, although they did not illustrate any time complexity analysis. He et al. [22] addressed a multi-task multi-instance synergistic deep learning strategy, named M2UNet for evaluation of the severity of corona features. They employed U-Net to segment the lung regions and lung lesions from the CT scan lung images. They achieved better performance in severity assessment for patients diseased by COVID-19. Chen et al. [23] presented some novel few-shot deep learning approaches for self-supervised analysis of COVID-19. They employed a contrastive learning strategy to train an encoder that can explore the animated feature representations on big pulmonary datasets and adjust the exemplary network for classification purpose. They also used stochastic data augmentation to render randomly example images into multiple views. Commencing with the justification of the instance discrimination to differentiate whether the two given images are similar illustrations or not, they generated multiple poses for the same images to supplement the original dataset. Then they employed self-supervised approach highlighted with a momentum contrastive learning strategy to further enhance the performance. They also put on the momentum mechanism to alleviate the local optima problem.

However, these existing approaches are trained with the fixed number of samples obtainable from a limited number of patients and sometimes are not capable of generalizing to new patients as deep learning strategies usually require a large amount of data for precise learning. A substantial number of research articles have been published on improving these issues. The convolutional neural networks (CNNs) like AlexNet [24], GoogleNet [25], MobileNetV2 [26], DenseNet [27], ResNet [28] and NasNetMobile [29] provide a classification task for COVID-19 features employing patients' CT scan images and they exhibit significantly high accuracy provided appropriate image enhancements are performed [30]. Abdulkareem et al. [31] trained three significant machine learning techniques like Navie Bayes, Random Forest, and support vector machine and applied Internet of Things (IoT) to diagnose patients with COVID-19 in smart hospitals. Based on laboratory dataset, they evaluated and recommended the most optimal diagnosis results among the selected ML models. Kumar et al. [32] employed a histogram based fast fuzzy C means clustering ROI extraction to detect lesion in COVID-19 CT images. They reduced the computational complexity compared to traditional fuzzy C means algorithm and produced auspicious outcome for 2D DICOM images. Dansana et al. [33] developed a convolutional network to diagnose COVID-19 infected patients earlier. They employed deep learning strategies like VGG-19, Inception_V2 and decision tree model instead of X-ray and CT scan image datasets.

This research addresses an image enhancement technique by shadowing pulmonary fibrosis, and crazy-paving pattern, air bronchogram, and halo sign using fuzzy expected value (FEV) for quality enhancement of the CT scan image captured for suspected coronavirus (COVID-19) patients. The approach is based on fuzzy histogram equalization, and it improves image contrast using the fuzzy normalized histogram of the input image. Experimental results indicate that this research improves the quality of the CT scan lung images using fuzzy expected value assessment and investigates the common imaging characteristics of lung in COVID-19 including lesions with GGO, lung consolidation, bilateral patch signs. These imaging interpretations provide not only for the detection and treatment of COVID-19 but also for the monitoring of disease progression and the assessment of therapeutic efficacy.

## 2. Materials and Methods

### 2.1. Image Enhancement over Fuzzy Expected Value Assessment

Image enhancement is performed with the idea of mapping the grayscale image into a fuzzy expected value plane, employing the membership functions. The membership function [34, 35] describes the characteristics of an image. The method is known as image fuzzification. The membershi*p* values are then modified in some manner to augment the contrast. The modified membership values are then inversely transformed through the procedure of defuzzification to generate an enhanced image. The fundamental steps involving in fuzzy enhancement algorithm are illustrated in Figure 1. The fuzzy expected value computation is accomplished with respect to the distance of each grey level from the corresponding fuzzy expected value.

### 2.2. Fuzzy Image Representation

A digital image I=*i* (*x*, *y*), consisting of *P* × *Q* pixels, is usually represented by a grid of pixels carrying light intensity or color information and stored in the matrix form. The traditional matrix notation is used to denote a digital image, where each matrix element is an ordered pair, (*i*(*x*, *y*), *μ*_*xy*_), where *i*(*x*, *y*) is the intensity of (*x*, *y*) positioned pixel and *μ*_*xy*_ is the membership degree of *i*(*x*, *y*). Thus the *P* × *Q* digital image is written in the following matrix form:

(1) $$\begin{array}{c} I=\left[\begin{array}{cccc} \left(i\left(0,0\right),\mu_{00}\right) & \left(i\left(0,1\right),\mu_{01}\right) & \cdots & \left(i\left(0,Y-1\right),\mu_{0X-1}\right)\\ \left(i\left(1,0\right),\mu_{10}\right) & \left(i\left(1,1\right),\mu_{11}\right) & \cdots & \left(i\left(1,Y-1\right),\mu_{1Y-1}\right)\\ \begin{array}{c} .\\ .\\ . \end{array} & \begin{array}{c} .\\ .\\ . \end{array} & \cdots & \begin{array}{c} .\\ .\\ . \end{array}\\ \left(i\left(X-1,0\right),\mu_{P-10}\right) & \left(i\left(X-1,1\right),\mu_{P-11}\right) & \cdots & \left(i\left(X-1,Y-1\right),\mu_{P-1Q-1}\right) \end{array}\right] \end{array}$$

where *P* is the number of rows and *Q* is the number of columns. The range of gray levels is [0, *G* − 1]. The membership degree of each intensity ranging [0, *G*-1] for each pixel of a classical image is either 0 or 1; i.e., *μ*_*xy*_ in equation (1) is either 0 or 1.

Fuzzy image is constructed based on fuzzy set theory, where each element of this set has some membership degree in the interval [0, 1]. The fuzzification of the gray levels is accomplished by the transformation function *ℑ* as follows:

(2) $$\begin{array}{c} \mu_{mn}=I\left[\left(i\left(x,y\right)\right.\right]={\left[1+\frac{I_{\max}-I_{\min}}{\delta }\right]}^{-\varepsilon } \end{array}$$

where *I*_min_ and *I*_max_ are the minimum and maximum gray levels, *δ* ∈ [0, 1] and *ε* ∈ {1, 2} are the denominational and exponential fuzzifiers which are chosen empirically depending on the degree of grayness.

The recursive modification of the membership is determined by using some characteristic function, which is called fuzzy membership function. Most of the prevailing membership functions are triangular function, trapezoidal function, *s*-shaped function, *z*-shaped function, *Π*−shaped function etc. This research uses *s*-shaped function, given by the following expression [36, 37]:

(3) $$\begin{array}{c} \mu_{xy}=\left\{\begin{array}{c} 0,\;i\left(x,y\right)<\alpha \\ 2{\left(\frac{I\left(x,y\right)-\alpha }{\gamma -\alpha }\right)}^{2},\;\alpha \leq i\left(x,y\right)\leq \beta \\ 1-2{\left(\frac{I\left(x,y\right)-\gamma }{\gamma -\alpha }\right)}^{2},\;\beta \leq i\left(x,y\right)\leq \gamma \\ 1,\;i\left(x,y\right)\geq \gamma \end{array}\right\} \end{array}$$

where *β* is the crossover point, *α* and *γ* are the left and right breakpoints, respectively, *γ* is the point where the height of the *s*-shaped curve is 1 and *α* = 2*β* − *γ*. The membership function is illustrated in Figure 2.

The membership function for the classical images is discrete. However, in fuzzy set, the membership function over [0,255] is gradually changing. For this reason, the fuzzy image based on fuzzy set theory is more suitable than the classical image based on classical set theory.

The fuzzy expectation of a discrete random variable *r*, (*r* ∈ *r*_1_, *r*_2_, *r*_3_, ⋯, *r*_*n*_) with respective fuzzy probabilities *F*(*r*_1_), *F*(*r*_2_), *F*(*r*_3_), ⋯*F*(*r*_*n*_) is defined by:

(4) $$\begin{array}{c} F_{E}\left(r\right)=\overset{n}{\underset{i=0}{\sum }}r_{i}F\left(r_{i}\right),\text{where}\overset{n}{\underset{i=0}{\sum }}F\left(r_{i}\right)=1. \end{array}$$

The fuzzy histogram of a fuzzy image with gray levels in the range [0, *G*-1] is *f*_*h*_(*s*_*r*_) = |*s*_*r*_|, where *s*_*r*_ is the *r*-th gray level. Again, the normalized fuzzy histogram is given by:

(5) $$\begin{array}{c} f_{h}\left(s_{r}\right)=\frac{\left|r^{th}\text{gray level}\right|}{\left|\text{gray level}\right|} \end{array}$$

which is also similar to fuzzy probability.

The fuzzy histogram equalization technique is based on the fuzzy normalized histogram of the image that is defined by:

(6) $$\begin{array}{c} f_{he}\left(s_{r}\right)=\overset{r}{\underset{i=0}{\sum }}f_{hs}\left(s_{i}\right)=\overset{r}{\underset{i=0}{\sum }}\frac{\left|i^{th}\text{gray level}\right|}{\left|\text{gray level}\right|},\text{where }r=0,1,2,\cdots G-1. \end{array}$$

### 2.3. Contrast Improvement Using Fuzzy Expected Value

The contrast improvement technique is based on the fuzzy expected value, which is described in the previous section. The algorithm is shown below:

### 2.4. FEV (Image I(x,Y))

This algorithm increases the contrast of given image *i* using the fuzzy expected value. Let the maximum gray level be *G* and *g*_*pq*_ is the gray level of (*p*,*q*)-th pixel.

Step1. Construct the fuzzy image of the given image *i* using the following equation.

(7) $$\begin{array}{c} \mu_{pq}=\frac{g_{pq}}{G} \end{array}$$

where *μ*_*pq*_ is the degree of membership of pixel (*p*,*q*) and g_pq_ is the grey level of the (*p*,*q*)-th pixel.

Step2. Construct the fuzzy histogram of the fuzzy image.

Step3. Compute the fuzzy expected intensity value, FE, using equation (4).

Step4. Determine the disparity of gray level, *d*_*pq*_ from FE using the following equation.

(8) $$\begin{array}{c} d_{pq}=\sqrt{\left|{F_{E}}^{2}-{g_{pq}}^{2}\right|} \end{array}$$

Step5. Generate a new gray level applying the following expression:

(9) $$\begin{array}{c} g_{pq}^{\prime }=\left\{\begin{array}{c} \max\left(0,F_{E}-d_{pq}\right)\text{if }g_{pq}<F_{E}\\ \min\left(G-1,F_{E}+d_{pq}\right)\text{if }g_{pq}>F_{E},\\ F_{E}\;otherwise \end{array}\right. \end{array}$$

Figure 3 shows the contrast improvement of a CT scan image using fuzzy expected value.

## 3. Results and Discussion

The effectiveness of the algorithm has been justified over several experiments on different publicly available datasets of chest CT images of COVID-19 affected patients [30]. A wide variety of CT image outcomes are observed that differ depending on the stage and severity of the pneumonia with associated co-morbidity.

This study was carried out retrospectively to analyze the chest CT findings on a dataset of 254 patients infected by COVID-19 during June - November 2020. This research had no potential risks for patients, and there were no direct relationships between researchers and patients. Patients with laboratory-confirmed COVID-19 (confirmed by a reverse transcription polymerase chain reaction, RTPCR) were considered as Covid positive case. CT images were autonomously studied by two expert radiologists having experience more than 12 years and blinded to the clinical data. The insertion criteria were patients who had undergone the first chest CT less than 5 days from illness onset and had not received any antiviral treatment. The exclusion criteria were the unsatisfactory quality of chest CT images for analysis. The study was accomplished according to the ideologies of the Helsinki Declaration.

According to the severity of pneumonia, the features of CT chest images focused the following aspects: (a) lesion distribution: both lungs, left or right lung; (b) lobes involved: upper, middle, and lower; (c) lesion location in lung parenchyma with their radiological findings: Ground Glass Opacity (GGO), consolidation, craze-paving pattern, stripes, air bronchogram, halo sign, and (d) other findings: mediastinal lymphadenopathy, pleural effusion, and interlobular septal thickening.

In general, the lesions in the lung are usually bilateral, the lower lobes are more commonly affected, and the right middle lobe is the least involved one. Again, the most common and the earliest finding are GGO, which is frequently designated as hazy and patchy opacity with peripheral, bilateral, and subpleural distribution. Consolidations feature typically exhibit after 10–12 days of appearing of symptoms, after the GGO findings. It is defined as an area of augmented attenuation visualize primarily in the subpleural and peripheral area that obscures the bronchial and vascular markings. It affects the lung by filling the alveoli with exudative or transudative fluid and blood [38]. It has been reported that there is high mortality in patients with consolidation and the incidence of this radiological finding is significantly higher in older patients than younger patients [39]. Furthermore, crazy paving is a sign of progressive disease where there is thickening of interlobular septa and intralobular lines superimposed on a background of GGO, resembling irregularly shaped paving stones. This sign also represents alveolar oedema and interstitial inflammation, and its appearance may indicate that the disease is in an advanced stage [40]. Again, it is the first CT sign to resolve in the absorptive stage while the consolidation and GGO may persist for up to 26 days [39]. Air bronchogram can be seen in both GGO and consolidation which is defined as air-filled bronchi with high density area. Air bronchogram is also a sign of advanced disease that can be noticed after the second week of symptom onset. Halo sign is defined as a condition in which GGO surrounds the central nodule or mass.

The outcome of the fuzzy expected value (FEV) image enhancement technique has been employed to chest CT images of COVID-19 pneumonia patients, as shown in Figure 4. Features are not clear for the first two column images, like A1-A2, B1-B2, C1-C2, D1-D2, and E1-E2 (*δ*=0.5 and *δ*=0.7, respectively). For the third column images A3, B3, C3, D3, and E3, the value of *δ* was chosen as 0.9 and the image features are more distinct. (A1-A3): GGO with consolidation involved in peripheral distribution was detected in the left upper lobe. (B1-B3): GGO with consolidation and reticulation were identified in a peripheral distribution in the right lower lobe. (C1-C3): Consolidation with peripheral distribution in the lower lobes of the lungs. (D1-D3): GGO with consolidation diffusely distributed in the bilateral lungs. Air bronchogram and crazy paving pattern detected on the background of GGO and consolidation. (E1-E3): GGO with consolidation detected in the bilateral lower lobes, distributed along the peribronchovascular bundle and subpleural regions.

Among the 254 patients, 81.89% had features on both lungs; 9.5% on the left lung; and 10.24% on the right lung. The predominantly affected lobe was the right lower lobe (79.53%). The distribution of COVID-19 infection in different lobes of two lungs and in individual lungs is shown in Figure 5. The distribution of the CT imaging features according to the lesion characteristics is shown in Figure 6. All 254 patients infected by COVID-19 pneumonia showed GGO, 83.5% showed consolidation, 63.8% showed crazy paving, 30.7% air bronchogram, 26% stripe, and other features were a few in percentage.

To assess the performance of the proposed fuzzy image enhancement algorithm, the following indices were considered:

Accuracy: Accuracy represents the degree of closeness to the true value and is expressed by:

(10) $$\begin{array}{c} Accuracy=\frac{TP+TN}{TP+TN+FP+FN} \end{array}$$

Sensitivity: Sensitivity indicates the true positive rate and is expressed by:

(11) $$\begin{array}{c} Sensitivity=\frac{TP}{TP+FN} \end{array}$$

Specificity: Specificity indicates the true negative rate and is represented by:

(12) $$\begin{array}{c} Specificity=\frac{TN}{TN+FP} \end{array}$$

Precision: Precision identifies the positive prediction value and is represented by:

(13) $$\begin{array}{c} Precision=\frac{TP}{TP+FP} \end{array}$$

where *TP* is true positive, means the ill person is correctly recognized as ill.

*FP* is false positive, which means the healthy person is wrongly recognized as ill.

*TN* is true negative, which means the healthy person is correctly recognized healthy.

*FN* is false negative, which means the ill person is wrongly recognized as healthy.

The proposed image enhancement method provided consistent accuracy of 94.6%, specificity of 92.5%, sensitivity of 84.1%, and precision of 96.7% for the chest CT imaging features for COVID-19 patients, which are quite reasonable, as shown in Figure 7.

The performance of the proposed method has been compared to the most influential traditional methods employed for image enhancement [40] in terms of their histograms, as shown in Figure 8. Although the histograms of the gamma corrected image (b2) and the image enhanced by histogram equalization (c2) exhibit brighter due to the higher intensity distribution at the brighter grey levels, but image distortion occurs in brighter regions owing to the inappropriate setting of gamma parameters for large pixel intensities. The FEV, on the contrary, surges the global contrast of the image by efficiently spreading out the most frequent intensity values depending on the membershi*p* value. That is why COVID-19 features like lesion are more distinct in the processed output CT images.

The objective performance of the algorithm has been evaluated employing three parameters: (i) entropy computation, (ii) Peak Signal -to-Noise Ratio (PSNR) measurement, and (iii) calculating the contrast index. Entropy was computed employing Shannon's law, given by:

(14) $$\begin{array}{c} Entropy=-\overset{I_{\max}}{\underset{x=1}{\sum }}h_{x}{Log}_{2}h_{x} \end{array}$$

where *I*max is the maximum intensity of the enhanced image.

The PSNR was calculated as the ratio of the peak enhanced to the original signal, expressed by:

(15) $$\begin{array}{c} PSNR=10{Log}_{10}\left(\frac{I_{\max}^{2}}{MSD}\right) \end{array}$$

(16) $$\begin{array}{c} MSD=\frac{1}{PQ}\overset{P}{\underset{x=1}{\sum }}\overset{Q}{\underset{y=1}{\sum }}{\left(I_{e}-I_{0}\right)}^{2} \end{array}$$

where **I**_**e**_ and **I**_**0**_ are the enhanced and original images, respectively.

The contrast index was measured as ratio of the contrast of the enhanced image and the original image, expressed as [41]:

(17) $$\begin{array}{c} \sigma \left(f\right)=\sqrt{\frac{1}{PQ-1}\overset{P}{\underset{x=1}{\sum }}\overset{Q}{\underset{y=1}{\sum }}\left(i\left(x,y\right)-PQ\right)} \end{array}$$

(18) $$\begin{array}{c} I_{C}=\frac{\sigma \left(I_{e}\right)}{\sigma \left(I_{0}\right)} \end{array}$$

The objective performance of this image enhancement algorithm has been compared with Pal-King [41], Modified Pal-King [42], Reshmalakshmi [43], and Patel [36] approaches, as shown in Table 1.

The major contributions of this research are:

- Address an image enhancement technique employing fuzzy expected value (FEV)
- Detect the COVID-19 pneumonia patients using CT scan images collected from different sources which include patients suffering from pneumonia and healthy people
- Identify different features of CT images of lung for COVID-19 patients like Ground-Glass Opacity (GGO), crazy paving, and consolidation
- Provide an image interpretation scheme for the monitoring of COVID-19 disease progression and the assessment of therapeutic efficacy

The main shortcoming associated with this research is data size. The data used for this investigation embrace CT scan images of 254 patients. The execution of this approach can be improved with a larger dataset. Additional experiments and investigations should be accompanied with laboratory findings from other areas to confirm these outcomes.

## 4. Conclusions

This paper outlines the imaging features of lung CT scans for patients with COVID-19 infection. Through this study, we introduced a fuzzy image enhancement approach for the accurate and precise diagnosis of infected lung parenchyma of COVID-19 patients and visualized different clinical features extracted from scan CT images. These features have been investigated and observed that they are complementary to each other. Compared to existing approaches, the proposed fuzzy image enhancement method provides significant improvements to optimize the performance depending on the parameters of membership functions. The traditional contrast enhancement methods are over-enhanced or under-enhanced due to mapping functions and that is why the lesions are not accurately identified even in high contrast CT images. The proposed method, on the contrary, offers fuzzily upgraded contrast images where all regions of the lung field are distinct, prominent, and well visualised to go for final diagnosis in radiological perspective. Moreover, the performance of this image enhancement algorithm in chest CT imaging features for COVID-19 patients are justified visually over histogram analysis and quantitatively over entropy, PSNR, and contrast index measures. Again, the objective performance of the algorithm was evaluated with three parameters like entropy, PSNR, and contrast index. Though CT imaging plays a vibrant role to calculate the volume of the lesions and diagnose the disease, this procedure will facilitate clear visualization of the infected organs. This fuzzy image enhancement approach will assist the clinicians to provide precise observation and monitor the disease progression as a selection tool for infected patients of COVID-19 pneumonia.

## Figures and Tables

**Figure 1:** Fundamental steps involved in fuzzy image enhancement process.

**Figure 2:** s-shaped membership function.

**Figure 3:** Contrast improvement of CT scan image (a) original image (b) enhanced image using fuzzy expected value.

**Figure 4:** Image enhancement over FEV for chest CT images of COVID-19 pneumonia patients.

**Figure 5:** Distribution of COVID-19 infection in different lobes of two lungs and in individual lung.

**Figure 6:** Feature Distribution of CT scan images according to lesion characteristics of COVID-19 Pneumonia.

**Figure 7:** Performance of the image enhancement algorithm in chest CT imaging features for COVID-19 patients.

**Figure 8:** CT images and their respective histograms.

**Table 1:** Comparison of different approaches for objective performance measures.

Approaches	Entropy	PSNR	Contrast index
Pal-King	4.41	19.27 dB	0.47
Modified Pal-King	4.62	21.36 dB	0.69
Reshmalakshmi	5.24	12.62 dB	1.12
Patel	5.47	13.35 dB	1.63
Proposed approach	5.61	14.86 dB	1.84

## Data Availability

Data is available from its original source as cited in the article. The dataset was anonymized by the dataset authors and all patient data were removed from radiological reports and DICOM images.
